# Autophagy-Related Genes in Atherosclerosis

**DOI:** 10.1155/2021/6402206

**Published:** 2021-07-02

**Authors:** Yuankun Chen, Ao Zeng, Shumiao He, Siqing He, Chunmei Li, Wenjie Mei, Qun Lu

**Affiliations:** ^1^School of Life Sciences and Biopharmaceutics, Guangdong Pharmaceutical University, Guangzhou, China; ^2^Guangdong Province Key Laboratory of Pharmaceutical Bioactive Substances, Guangdong Pharmaceutical University, Guangzhou, China; ^3^Guangdong Province Engineering and Technology Center for Molecular Probe and Bio-medicine Imaging, Guangzhou, China

## Abstract

**Background:**

Atherosclerosis (AS) is a common chronic vascular inflammatory disease and one of the main causes of cardiovascular/cerebrovascular diseases (CVDs). Autophagy-related genes (ARGs) play a crucial part in pathophysiological processes of AS. However, the expression profile of ARGs has rarely been adopted to explore the relationship between autophagy and AS. Therefore, using the expression profile of ARGs to explore the relationship between autophagy and AS may provide new insights for the treatment of CVDs.

**Methods:**

The differentially expressed ARGs of the GSE57691 dataset were obtained from the Human Autophagy Database (HADb) and the Gene Expression Omnibus (GEO) database, and the GSE57691 dataset contains 9 aortic atheroma tissues and 10 normal aortic tissues. The differentially expressed ARGs of the GSE57691 dataset were analyzed by protein-protein interaction (PPI), gene ontology analysis (GO), and Kyoto Encyclopedia of Genes and Genomes analysis (KEGG) and were chosen to explore related miRNAs/transcriptional factors.

**Results:**

The GSE57691 dataset had a total of 41 differentially expressed ARGs. The GO analysis results revealed that ARGs were mainly enriched in autophagy, autophagosome, and protein serine/threonine kinase activity. KEGG analysis results showed that ARGs were mainly enriched in autophagy-animal and longevity regulating signaling pathways. Expressions of ATG5, MAP1LC3B, MAPK3, MAPK8, and RB1CC1 were regarded as focus in the PPI regulatory networks. Furthermore, 11 related miRNAs and 6 related transcription factors were obtained by miRNAs/transcription factor target network analysis.

**Conclusions:**

Autophagy and ARGs may play a vital role in regulating the pathophysiology of AS.

## 1. Introduction

Autophagy, a capacity of maintaining cellular homeostasis, is a process of damaging cytosolic material and delivering to lysosomes for degradation, leading to the turnover of cell material and providing macromolecular precursors [1, 2]. Autophagy deficiency is closely related to multiple diseases, such as cancers, CVDs, and immune disorders [3, 4].

CVDs still remain a prevalent cause of mortality and morbidity worldwide, affecting 16.7 millions of individuals each year [5]. One of main causes of acute cardiovascular death is AS. AS is a common chronic inflammatory disease characterized by atherosclerotic plaque and vascular stenosis [6, 7].

Studies have shown that autophagy may be involved in regulating cell survival and death during the occurrence and development of AS [8, 9]. In the early stage of atherosclerotic lesions, autophagy can inhibit the apoptosis of vascular endothelial cells and delay the development of atherosclerotic plaques. In the late stage of atherosclerotic lesions, excessive activation of autophagy leads to autophagic death of vascular cells, decreased collagen synthesis, and weak fibrous caps that cause plaque rupture. Vascular smooth muscle cells (VSMCs) play a significant role in atherogenesis. Autophagy in VSMCs protects cells in AS plaque by suppressing oxidative stress, inhibiting mitochondrial depolarization and degrading damaged substances [10]. Furthermore, successful autophagy inhibits VSMCs senescence, whereas defective autophagy accelerates atherogenesis. The role of autophagy in AS remains undefined though a series of studies have reported that autophagy is activated in AS.

In the past few years, bioinformatics and microarray technologies have been widely used to excavate the genetic targets of multiple diseases, which have helped researchers in identifying the differentially expressed genes and potentially different signaling pathways. However, few research studies applied to explore the relationship between autophagy and AS.

In this study, we used ARGs to explore the relationship between AS and autophagy. The differentially expressed ARGs were screened, and the relevant data were processed by GO and KEGG analysis. The complex interaction between miRNAs/transcriptional factors and genes was predicted. This main aim of study is to explore the relationship between autophagy and AS.

## 2. Methods

### 2.1. Data Collection

A total of 232 ARGs were gathered from the HADb (http://www.autophagy.lu/index.html) [11]. GEO (http://www.ncbi.nlm.nih.gov/geo) is a high-throughput resource functional genomics database that includes chips, microarrays, and gene expression data [12]. GSE57691 dataset was obtained from the GEO database, which contains 9 aortic atheroma tissues and 10 normal aortic tissues. Meanwhile, the probe is converted into a homologous gene symbol using the annotation information on the platform.

### 2.2. Differentially Expressed ARGs

The limma method in *R* was used to analyze the differential expression of ARGs between the AS group and control group [13]. The threshold was the adjusted *P* value <0.05 and | log2 fold change (FC) |>2 [14].

### 2.3. Data Repeatability Test

The intragroup data repeatability of each group was verified by Pearson's correlation. *R* programming language provides operating environment and software for drawing of graphs and statistical analysis [15]. Use heatmaps to visualize correlations between samples in the same dataset and using *R* to draw the heatmap. Principal component analysis (PCA) is a sample clustering method for gene expression, diversity analysis, and resequencing [16]. The sample cluster analysis method is used to verify the intragroup data repeatability of the dataset.

### 2.4. GO and KEGG Online Enrichment Analysis

The enrichment analysis of GO [17] and KEGG [18] in ARGs were performed through DAVID (version 6.8, Database for Annotation, Visualization, and Integrated Discovery, https://david.ncifcrf.gov/) [19]. The visual GO and KEGG enrichment plots of annotation results were analyzed through “digest” and “GO plot” packages in *R* [20].

### 2.5. PPI Regulatory Network Construction

Evaluate the interaction between ARGs through the STRING database (version 11.0, https://string-db.org/) [21]. In addition, a combined score >0.4 was considered to be a statistically significant interaction. Then, the PPI regulatory network analysis results are loaded into Cytoscape for visualization [22, 23].

### 2.6. miRNAs/Transcription Factor Networks Construction

The miRNAs/transcription factor was analyzed by WebGestalt (http://www.webgestalt.org/) [24]. The correlation between the miRNA/transcription factor and ARGs in significant clustered modules was analyzed by overrepresentation enrichment analysis (http://amp.pharm.mssm.edu/Enrichr/) [25]. Finally, Cytoscape was used to visualize the miRNAs/transcription factor network [24].

## 3. Results

### 3.1. Repeatability Verification of Dataset

We used the PCA and Pearson's correlation test to validate the GSE57691 dataset repeatability. According to the PCA, the intragroup repeatability of the GSE57691 dataset was acceptable. In the control group and the AS group, the distances between per sample were close in the dimension of principal component 1. In addition, the distances between the control group and the AS group were far (Figure 1(b)). Pearson's correlation test revealed that there was a strong correlation among the samples in the control group and there was a strong correlation among the samples in the AS group of the GSE57691 dataset. Moreover, sample in the control group and sample in the AS group exist a negative correlation (Figure 1(a)).

### 3.2. Differentially Expressed ARGs Identified between the AS Group and Control Group

In the GSE57691 dataset, 41 differentially expressed ARGs, including 20 upregulated ARGs (TBK1, BID, GNAI3, PTK6, and so on) and 21 downregulated ARGs (ITGA3, WIPI2, MAPK3, FADD, and so on), were identified in the AS group, as shown in heatmap (Figure 2(a)). In addition, the differentially expressed ARGs between the control group and AS group are shown in volcano plot (Figure 2(b)).

### 3.3. Functional and Pathway of Differentially Expressed ARGs Enrichment Analysis

Based on the GO analysis, we found that the biological processes of differentially expressed ARGs were markedly enriched in autophagy, process utilizing autophagic mechanism, and macroautophagy. The cell components of differentially expressed ARGs were markedly enriched in autophagosome, vacuolar membrane, and phagophore assembly site membrane. The molecular function of differentially expressed ARGs was markedly enriched in protein serine/threonine kinase activity, MAP kinase activity, and ubiquitin protein ligase binding (Figure 3(a)). The results of the KEGG analysis showed that differentially expressed ARGs were primarily enriched in the autophagy-animal signaling pathway and longevity regulating signaling pathway (Figure 3(b)).

### 3.4. PPI Regulatory Network and Module Analysis, Hub Gene Identification and Analysis

The PPI regulatory network of differentially expressed ARGs was constructed (Figure 4(a)). The PPI regulatory networks contain 35 nodes and 135 interacting pairs. Then, the most significant module and hub genes in the network were screened by Cytoscape (Figures 4(b) and 4(c)). A total of 10 hub genes with degrees ≥13 were screened: PTEN, FOXO3, RPS6KB1, MAP1LC3A, ULK1, RB1CC1, MAPK8, MAPK3, MAP1LC3B, and ATG5. In addition, subnet modules A and B were selected in the PPI regulatory network. Module A contains 6 upregulated nodes (WDFY3, ATF4, ATG4D, and so on), 10 downregulated nodes (MAP1LC3A, MAPK3, MAPK8, and so on), and 56 interacting pairs. Module B contains 3 upregulated nodes (HSPAB, RB1CC1, and ATG5), 1 downregulated nodes (MAP1LC3A), and 5 interacting pairs. The genes in the two modules are given in Table 1.

### 3.5. miRNAs/Transcription Factor Target Networks Analysis

11 miRNAs (miR-181 family had the most targets) and 6 transcription factors (CREB, ATF, FREAC2, ATF3, CREBP1CJUN, and AP1) were predicted, and 92 regulatory pairs of miRNA and transcription factor networks were constructed (Figure 5). There were 13 upregulated genes and 16 downregulated genes in the miRNAs/transcription factor networks. In the miRNA networks, 13 regulatory interactions were found between upregulated genes and miRNA, and 16 regulatory pairs were identified between downregulated genes and miRNA. In the transcription factor networks, FREAC2 was predicted to target 3 upregulatory genes (CDKN1B, FOXO1, and GRID2) and 5 downregulatory genes (FOXO3, KLHL24, MAPK3, ULK1, and WIPI2). CREB was predicted to target 3 upregulatory genes (ATG5, EEF2, and ST13) and 2 downregulatory genes (MAP1LC3A and RAB24).

## 4. Discussion

Mounting evidence indicates that autophagy participates in maintaining cardiovascular health. Dysfunction of vascular autophagy is related to the initiation of CVDs [26]. Additionally, ARGs affect AS through regulation of VSMCs phenotypic switching, lipid metabolism, and other biological processes [27, 28].

Gene microarray technology is a new method to explore new biomarkers of diseases. Huang et al. screened 98 differentially expressed genes from AS macrophages through DNA microarray analysis and then identified KDELR3, CD55, and DYNC2H1 as key genes through a series of analysis [29]. Another study predicted that miR-126 may be a biomarker of AS through gene microarray technology, and its overexpression may prevent the occurrence and development of AS. In addition, lncRNA microarray was also used to study AS. LncRNA-FA2H-2 may improve AS by affecting autophagy and inflammation [28].

In the current study, in order to determine the relationship between ARGs and AS, microarray analysis was used to identify differentially expressed ARGs from the AS group and the control group. First, we screened 41 differentially expressed ARGs between the AS group and control group. Based on GO and KEGG analysis, we found that differentially expressed ARGs involve multiple biological processes and signaling pathways, including autophagy, autophagosome, and autophagy-animal signaling pathway. Then, a total of 10 hub genes (PTEN, FOXO3, RPS6KB1, MAP1LC3A, ULK1, RB1CC1, MAPK8, MAPK3, MAP1LC3B, and ATG5) were identified through the PPI regulatory network. Finally, the miRNAs/transcription factor networks were constructed, including 11 miRNAs and 6 transcription factors.

In the BP analysis, most genes were enriched in autophagy. Osonoi et al. found that the degree of autophagy increased in the atherosclerotic smooth muscle cells of human and rabbit by transmission electron microscopy [30]. In the CC analysis, most genes were enriched in autophagosome. The main role of autophagosomes is to transfer organelles and proteins to lysosomes for degradation. Zhang et al. reported that CAV-1 controls autophagic flux and the formation of autophagosomes by affecting the cellular localization of autophagosomes in lipid rafts, thus influencing the development of AS [31]. In the MF analysis, protein serine/threonine kinase activity enriched the most genes. AKT, the downstream target of PI3K, is serine/threonine protein kinase. PI3K/AKT is one of the main pathways of autophagy regulation. Previous studies have reported that Shen-Yuan-Dan capsule treatment reduces foam cell formation by activating autophagy via affecting the PI3K/AKT/mTORC1 signaling pathway [32]. The KEGG analysis showed that the autophagy-animal signaling pathway might play a role in AS-related autophagy. The AMPK signaling pathway and mTOR signaling pathway are two major pathways in the autophagy-animal pathway. Wu et al. reported that paeonol inhibits the excessive proliferation of VSMCs by inducing AMPK phosphorylation, reducing mTOR phosphorylation, and upregulating autophagy [33].

A total of 10 hub targets were identified in the PPI regulatory network, including ATG5, MAP1LC3B, MAPK3, MAPK8, and RB1CC1. Previous study reported that ATG5 is involved in autophagosomes formation [34]. In addition, ursolic acid exerted antiatherosclerosis effects and protected human umbilical vein endothelial cells (HUVECs) from ox-LDL induced cytotoxicity. The underlying mechanism is associated with increased SIRT1 expression, reduced acetylation of lysine residue on Atg5, and enhanced autophagy [35]. These suggest that ATG5 may play an important role in autophagy associated with AS. MAP1LC3B is indirectly related to plaque instability, which may prevent atherosclerotic plaque instability by promoting basic autophagy activity. Meanwhile, Bhairavi Swaminathan et al. found that low expression of MAP1LC3B in carotid atherosclerotic plaques did not induce related autophagy. This may cause dead cells to accumulate at the site of the lesion and subsequently lead to cerebrovascular events [36]. MAPK3 (ERK1) and MAPK8 (JNK1) are members of the mitogen-activated protein kinase family (MAPK). MAPK signaling pathway plays a vital role in the pathogenesis of CVDs [37]. Babaev et al. found that the reduction of JNK1 in macrophages protects them from apoptosis and increases cell survival rate, thus accelerating early AS [38]. In addition, Zheng et al. reported that protocatechuic acid improved vulnerable lesions in mice, which may be caused by the upregulation of MERTK to normalize arterial inflammation and inhibit MAPK3/1 in lesional macrophages [39]. RB1CC1 is involved in the composition of ULK1-ATG13-RB1CC1/RB1CC1-ATG101 complex, which is crucial for the formation of autophagosome [40, 41]. RB1CC1 is also involved in protein synthesis, cell proliferation and migration, differentiation, and cell cycle processes [42]. However, RB1CC1 is rarely reported on CVDs.

Based on the analysis of miRNAs/transcription factor target networks, we found that miR-506 had 7 targeted ARGs, which exerted the most obvious target interaction among the 10 analyzed miRNAs. In particular, miR-506 regulates the hub gene RB1CC1, and the highly expressed RB1CCI in the network is downregulated by miR-506. RB1CC1 is essential for the formation of autophagosomes. In addition, the low expression of CAPN1 in the network was upregulated by miR-506. Calpain is involved in inflammation and AS [43]. Yin et al. reported that the downregulation of Calpain-1 and inactivation of Calpain might be closely related to the anti-inflammatory and antiatherosclerosis effects of simvastatin [44]. Therefore, the axes of miR-506-CAPN1 and miR-506-RB1CC1 may be closely related to AS and autophagy [45, 46].

## 5. Conclusion

In summary, our current study has evaluated the expression of ARGs in AS based on the GEO database and HADb. We found that ARGs were involved in the occurrence and development of AS through multiple biological processes and signaling pathways, such as autophagy, process utilizing autophagic mechanism, macroautophagy, and autophagy-animal signaling pathway. In addition, we also found that the axes of miR-506-CAPN1 and miR-506-RB1CC1 may be closely related to AS and autophagy. Taken all of these, ARGs may play a vital role in AS.

## Figures and Tables

**Figure 1:** Intragroup data repeatability of the GSE57691 dataset verified by Pearson's correlation and PCA analysis. (a) Pearson's correlation analysis of intragroup data from the GSE57691 dataset. The color represents the degree of correlation. 0< correlation <1 indicates a positive correlation, and −1< correlation <0 indicates a negative correlation. When the absolute value of a number is large, there exists a strong correlation. (b) PCA analysis of intragroup data from the GSE57691 dataset. In the scatter diagram, PC1 and PC2 represent *X*-axis and *Y*-axis, respectively, where each point is a sample. The distance between the two samples represent the difference in gene expression patterns.

**Figure 2:** Differential expressions of ARGs between the control group and AS group. (a) The 41 differentially expressed ARGs from the GSE57691 dataset. *C* indicates the control group and *T* indicates the AS group. (b) Volcano plot of differentially expressed ARGs. Red indicates high expression genes, green indicates low expression genes, and black indicates that there is no difference in these genes between the AS group and control group.

**Figure 3:** GO and KEGG enrichment analysis of 41 differentially expressed ARGs. (a) Histogram of GO enrichment. (b) Histogram of KEGG enrichment.

**Figure 4:** PPI regulatory network and subnet module analysis of differentially expressed ARGs. The nodes represent the ARGs, and the lines indicate the interaction of two ARGs. The size and color of nodes are positively correlated with the degree and closeness centrality. (a) PPI regulatory networks. (b), (c) Subnet module analysis of PPI regulatory networks.

**Figure 5:** miRNAs/transcription factor target networks. The red circles indicate the upregulated ARGs, and the green circles indicate the downregulated ARGs. The violet triangle indicates miRNAs, and the yellow quadrilateral indicates transcription factors.

**Table 1:** Submodule ARGs and degree of PPI regulatory networks.

Module A			Module B		
Node	Description	Degree	Node	Description	Degree
WDFY3	Up	8	HSPA8	Up	9
ATG4D	Up	8	RB1CC1	Up	15
CDKN1B	Up	8	MAP1LC3B	Down	19
ATG4A	Down	9	ATG5	Up	22
ATF4	Up	9
FOXO1	Up	10
WIPI2	Down	11
LAMP2	Up	11
ATG14	Down	12
PTEN	Down	13
FOXO3	Down	13
RPS6KB1	Down	14
MAP1LC3A	Down	14
ULK1	Down	14
MAPK8	Down	16
MAPK3	Down	18

## Data Availability

The data used to support the findings of this study have not been made available because authors were not given permission to share the data.
